RETRACTED

# Silver Nanoparticles Stabilized by Poly (Vinyl Pyrrolidone) with Potential Anticancer Activity towards Prostate Cancer

**DOI:** 10.1155/2022/6181448

**Published:** 2022-09-30

**Authors:** Ahmed A. H. Abdellatif, Ahmed Abdelfattah, Abdellatif Bouazzaoui, Shaaban K. Osman, Issa Saad Al-Moraya, Abdulaziz M. Saleh Showail, Mansour Alsharidah, Ashraf Aboelela, Osamah Al Rugaie, Tarek M. Faris, Hesham M. Tawfeek

**Affiliations:** ^1^Department of Pharmaceutics, College of Pharmacy, Qassim University, Buraydah, Qassim 51452, Saudi Arabia; ^2^Department of Pharmaceutics and Pharmaceutical Technology, Faculty of Pharmacy, Al-Azhar University, Assiut 71524, Egypt; ^3^Department of Industrial Pharmacy, Faculty of Pharmacy, Assiut University, Assiut, Egypt; ^4^Department of Medical Genetics, Faculty of Medicine, Umm Al-Qura University, Makkah 21955, Saudi Arabia; ^5^Science and Technology Unit, Umm Al-Qura University, Makkah 21955, Saudi Arabia; ^6^Medical Clinic, Hematology, Oncology, University Hospital Regensburg, Franz-Josef-Strauß-Allee 11, Regensburg 93053, Germany; ^7^Clinical Toxicology, College of Medicine Umm Al-Qura University, Makkah 21955, Saudi Arabia; ^8^Forensic Medicine & Toxicology Center, Ministry of Health, Abha, Saudi Arabia; ^9^Department of Urology, Khamis Mushait General Hospital, Ministry of Health, Khamis Mushait, Saudi Arabia; ^10^Department of Physiology, College of Medicine, Qassim University, Buraydah 51452, Saudi Arabia; ^11^Department of Pharmaceutical Chemistry, Faculty of Pharmacy, Sphinx University, Assiut, Egypt; ^12^Department of Basic Medical Sciences, College of Medicine and Medical Sciences, Qassim University, Unaizah, P.O. Box 991, Al Qassim 51911, Saudi Arabia; ^13^Department of Pharmaceutics and Industrial Pharmacy, College of Pharmacy, Al-Azhar University, Cairo 11884, Egypt

## Abstract

Tumor necrosis factor (TNF-*α*) and inflammatory cytokine (IL-6) play a vital role in various cellular incidents such as the proliferation and death of cells during carcinogenesis. Hence, regulation of these biomarkers could be a promising tool for controlling tumor progression using nanoformulations. Silver nanoparticles-poly (vinyl pyrrolidone) (AgNPs-PVP) were prepared using the reduction of silver nitrate and stabilized with PVP. They are characterized through yield percentage, UV-VIS, FT-IR, size, charge, and morphology. The obtained AgNPs were tested for anticancer activity against prostate cancer (PC 3) and human skin fibroblast (HFS) cell lines. Moreover, biomarker-based confirmations like TNF-*α* and IL-6 were estimated. The synthesized AgNPs-PVP were stable, spherical in shape, with particle sizes of 122.33 ± 17.61 nm, a polydispersity index of 0.49 ± 0.07, and a negative surface charge of −19.23 ± 0.61 mV. *In vitro* cytotoxicity testing showed the AgNPs-PVP exhibited antiproliferation properties in PC3 in a dose-dependent manner. In addition, when compared to control cells, AgNPs-PVP has lower TNF-*α* with a significant value (^*∗*^*p* < 0.05); the value reached 16.84 ± 0.71 pg/ml versus 20.81 ± 0.44 pg/ml, respectively. In addition, HSF cells showed a high level of reduction (^*∗∗∗*^*p* < 0.001) in IL-6 production. This study suggested that AgNPs-PVP could be a possible therapeutic agent for human prostate cancer and anti-IL-6 in cancerous and noncancerous cells. Further studies will be performed to investigate the effect of AgNPs-PVP in different types of cancer.

RETRACTED

## 1. Introduction

Cancer is still among the most common and deadly diseases worldwide. The latest investigations conducted by the National Cancer Institute showed almost 18.1 million new cases and 9.5 million deaths worldwide as recorded in 2018 related to cancer. This number is set to reach 29.5 million cases in 2040 [1]. A lot of research and investigations have been performed to prepare an effective and safe medication for patients suffering from cancer. Prostate cancer in men is considered one of the most known tumors that significantly affect men's reproductive systems [2]. Hence, rapid diagnosis and effective therapy are the essential issues. It is also expected to spread to 24 million cases by 2035 [3]. Surgical intervention via prostatectomy can terminate the problem. However, in some cases, surgical removal is not sufficient, and the recurrence of the tumor is often diagnosed.

The era of nanomedicine and nanoparticulate drug delivery systems has begun long ago and shown significant success in different fields, especially tumor diagnosis and treatment [4–9]. Nanoparticles directed at cancer have been shown to be promising materials in this area. Their unique physicochemical properties have enabled them to deliver different anticancer drugs and other molecules like genes via active and passive targeting [9–12]. Recently, Almowalad et al. studied the efficiency of lactoferrin-bearing gold nanocages for gene delivery in prostate cancer *in vitro*. The authors found that lactoferrin-bearing gold nanocages alone or conjugated with polyethyleneimine and polyethylene glycol were able to condense DNA at conjugate DNA weight ratios of 10 : 1 and even higher ratios due to enhanced DNA cellular uptake [13, 14].

Metallic NPs appear as promising nanomaterials for efficient anticancer activity, e.g., gold, silver, and quantum dots [7, 14, 15]. Abaza et al. examined the antitumor activity of a chitosan/polyvinyl alcohol blend doped with gold and silver NPs in the treatment of a prostate cancer model. They further concluded their findings with a significant antitumor effect against prostate cancer [16].

RETRACTED

Silver nanoparticles (AgNPs) hold a significant effect on cancer therapy due to cancer-specific selectivity, low side effects, and massive anticancer activities [17]. Chen et al. explored the role and mechanism of AgNPs in prostate cancer. The authors reported that AgNPs affect the integrity of the lysozyme membrane and cause a lowering in their number and attenuation of lysosomal protease activity. Such activity resulted in a blockage of autophagic flux. In addition, using sublethal doses of AgNPs could induce hypoxia and energy deficiency in PC-3 cell lines [18]. Saravan Kumar and Wang synthetized biogenic AgNPs embedded with magnesium oxide NPs. A cytotoxicity study showed that the combined NPs system caused more substantial cell death in the prostate cancer cell line PC-3 than magnesium oxide NPs alone [19]. AgNPs have represented significant anticancer activity against different types of malignancies, such as prostate [2], lung [20], leukemia [21], cervical [22], hepatic [23], colorectal [24], and breast [25].

Firdhouse and Lalitha successfully synthesized ultrafine AgNPs using a green approach. The produced nanosilver showed anticancer activity against PC3. In addition, the biosynthesis of AgNPs can be an alternative to the traditional method of synthesis [26]. AgNPs can be prepared in different ways [27] through chemical, physical, and biological means. Afterward, they showed aggregations that can be prevented using different stabilizers, such as cellulosic polymers [28] and chitosan [29].

A previous study in our research group has demonstrated the antitumor activity of AgNPs prepared using ethyl cellulose as a reducing and stabilizing agent. AgNPs were efficiently produced with high stability, and they inhibited TNF-*α* in breast cancer cell lines. In addition, AgNPs exerted an inhibitory effect on cytokine mRNA and protein expression levels [7]. Tumor necrosis factor, TNF-*α*, which is also known as lipopolysaccharide, is secreted by malignant epithelial cells found in different malignant tissues [30, 31]. It could promote tumor cell migration and invasion via autocrine surviving signals for tumor cells. Furthermore, they regulate the infiltration of tumor-promoting macrophages into the tumor microenvironment [32]. Interleukin IL-6, as an inflammatory cytokine, has been shown to be a major regulator of prostate cancer progression [33]. During the carcinogenesis process, inflammation could affect this process at the molecular level by regulating the tumor microenvironment through the alteration of the balance of cytokines, chemokines, transcriptional factors, and reactive oxygen species [34]. TNF-*α* and IL-6 have been shown to be associated with prostate cancer progression [35]. IL-6 and TNF-*α* are two cytokines with multiple and overlapping biological properties, that are involved in the development of prostate cancer [36, 37]. Studies of IL-6 in prostate carcinoma provide support for the hypothesis that direct local production of IL-6 by malignant cells significantly contributes to elevated serum levels [38]. This study aimed to investigate the utilization of polyvinyl pyrrolidone, or PVP, as a reducing agent and stabilizer for stabilized dispersion of AgNPs. In addition, the effect of these NPs on the prostate cancer cell line PC-3 was also studied. The expression levels of TNF-*α* and IL-6 were also measured to gain a better understanding of the role of these NPs in prostate tumor inhibition or regression.

RETRACTED

## 2. Materials and Methods

### 2.1. Materials

Silver nitrate was purchased from VBBN Company, Hong Kong, China. PVP K25 was obtained from Sigma-Aldrich, UK. Human skin fibroblasts, HSF, prostate cancer cell lines, PC3, ATCC, Manassas, VA, USA. Media DMEM, Lonza Bioscience, Switzerland. Penicillin, streptomycin, fetal bovine serum albumin, and MTT assay kit (Sigma-Aldrich, Taufkirchen, Germany). Deionized water was used throughout the study and secured using a Milli-Q® water purifier (Millipore, France).

### 2.2. Methods

#### 2.2.1. Preparation of AgNPs-PVP

AgNPs stabilized with PVP were prepared as previously published with our research group [28]. Briefly, a stock of 1% w/v PVP in aqueous solution was prepared. 2 ml of PVP solution was dropped into 100 ml of AgNO_3_ 1 mM aqueous solution and heated to 100°C with stirring. The solution color turned brownish-green, indicating the formation of AgNPs-PVP. Afterward, the heating was terminated, and the solution was stirred until it got cold. The obtained cold solution was filtered via centrifugation for 7 min at 1500 rpm. The collected precipitate was discarded. The clear supernatant was stored in the fridge at 7–10°C as a purified AgNPs-PVP for further characterization.

### 2.3. Characterization of AgNPs-PVP

#### 2.3.1. Percentage Yield of the Prepared AgNPs

The number of silver cations converted to silver metal was calculated as an indication of the percent yield of the produced AgNPs. Briefly, samples were diluted with five percent nitric acid to facilitate the detection of silver (free, unreacted, and reacted) at the selected, wavelength of 324 nm. Unreacted silver cations were precipitated from sample solutions via the addition of sodium chloride solution leaving silver cations soluble in the solution. The formed silver chloride precipitate was then removed via centrifugation at 2000 rpm for 15 min. The supernatant was analyzed for silver cations using inductively coupled plasma optical emission spectrometry (ICP-OES, iCAP 6000, Thermo Scientific, USA). Then, the AgNPs yield percentage was calculated using the following equation [28, 39].

(1) $$\begin{array}{c} \%\text{AgNPs yield}=\left[\frac{\text{concentration of each sample by ICP}-\text{OES}}{\text{initial}c\text{oncentration of }{\text{AgNO}}_{3}}\right]\times 100. \end{array}$$

RETRACTED

#### 2.3.2. UV-VIS Spectroscopy

The AgNPs-PVP solution was scanned from 300 to 600 nm using a UV-VIS spectrophotometer (Lambda 25, Perkin Elmer, Singapore). The UV-VIS absorption was performed after centrifugation of the obtained AgNPs-PVP particles, followed by redispersion of the obtained pellets in distilled water [40].

#### 2.3.3. Fourier-Transform Infrared Spectroscopy (FT-IR)

An FT-IR study was performed using an FT-IR spectrometer (Alpha II, model: Bruker, USA). Simply, PVP, AgNO_3,_ and AgNPs-PVP solutions were investigated for interactions and computability as well as to get proof of polymer coating via observing the collected spectra obtained after their scanning from 4000–400 cm^−1^ [41].

#### 2.3.4. Transmission Electron Microscopy

TEM was used to observe the morphology of the produced AgNPs-PVP and to measure the diameter of the particles. Briefly, 10 *μ*l of each AgNPs-PVP solution was applied to the surface of the double-sided copper conductive tape and allowed to dry overnight [42]. Afterward, nanoparticles were viewed under the microscope at 10–100 *k* magnification power using an accelerating voltage of 100 kV. (JEM-1230, Joel Japan).

#### 2.3.5. Size and *ζ* Potential

A Zetasizer Nano particle size analyzer was used to investigate the geometrical particle size of the produced AgNPs. An aqueous solution of each sample was adjusted to ≈25°C and then exposed to a laser beam of ≈633 nm at a scattering angle of ≈90°. The obtained results were calculated as the average of the three measurements, whereas each measurement was run ≈20 times (with *a*≈10 s duration) [43]. Furthermore, the *ζ* potentials (*ζ*) of all formulated AgNPs were determined using a Malvern Zetasizer Nano ZS Malvern Instruments (Malvern, UK).

### 2.4. Physical Stability

The physical stability of the prepared AgNPs-PVP was investigated at two different storage conditions (25.0 ± 0.5°C and 4.0 ± 0.5°C) for a period of 3 months. The physical appearance of NPs, including their color, morphology, particle size, and zeta potential, were investigated at the beginning and after the storage period to make sure of the particle's stability towards aggregation and the suitability of PVP to produce a homogeneous dispersion.

RETRACTED

### 2.5. Cell Culture

In this study, PC3 and HSF cell lines were chosen. The PC3 cells have been cultivated in an F-12K medium supplemented with 10% heat-inactivated fetal bovine serum (FBS) and 1% penicillin/streptomycin purchased from Invitrogen (Thermo Fisher Scientific, Karlsruhe, Germany). The HSF was maintained in DMEM media supplemented with 10% heat-inactivated FBS and 1% of penicillin/streptomycin. Both types of cells were incubated at 37°C and 5% CO_2_ [44].

### 2.6. MTT Cytotoxicity Assay

The cytotoxicity of the AgNPs/PVP as well as PVP and AgNO_3_ were tested on HSF and PC3 cells using the (3-(4, 5-dimethylthiazolyl-2)-2, 5-diphenyltetrazolium bromide (MTT) assay. In the test, the mitochondria of viable cells change hydrophilic tetrazolium salt (yellow color) into a hydrophobic purple dye known as formazan, and the strength of the color correlates with the number of surviving cells [45].

The MTT test was conducted as previously described [44]. On the first day, the cells were suspended at a density of 1.2–1.5 × 10^4^ cells/mL in 100 *μ*L suitable media and were seeded into each well of the 96-wells microtiter plate and incubated for 24 h. The next day, the formulations were dissolved in 0.5% DMSO, passed through 0.450 *μ*m syringe filters, and added to the wells in triplicate at the corresponding concentrations. For the HSF cells, concentrations of 0.5, 5, 50, 500, and 5000 *μ*g/ml of the PVP aqueous solution were evaluated. For AgNPs/PVP and AgNO_3_ aqueous solutions, concentrations from 0.4–100 *μ*g/ml were investigated. Thereafter, cells were incubated at 37°C with 5% CO_2_ for 24 h. The next day, the media were replaced with fresh ones and a standard MTT assay was conducted according to the manufacturer's instructions. Briefly, 100 *μ*l of 5 mg/ml MTT in the medium was added to the cells and incubated for 4 hours at 37°C with 5% CO_2_. After that, the formulated formazan crystals were dissolved in 100 *μ*l of 1% HCl in Isopropanol, and the absorbance of each sample was measured at 570 nm using a microplate reader (BioTek, Winooski, VT, USA). The inhibitory concentration was estimated at 50% (IC_50_) from an exponential viability curve versus the norms' concentration.

Cell viability was determined by Equation (2).

(2) $$\begin{array}{c} \text{cell }v\text{iability\%}=\frac{{\text{absorbance}}_{\text{sample}}\;}{{\text{absorbance}}_{\text{control}}}\;\times 100. \end{array}$$

### 2.7. TNF and IL6 Enzyme-Linked Immunosorbent Assays (ELISA)

To test the effect of the different formulations on TNF and IL6 production in the cells, 1.5 × 10^4^ PC3 or HSF/mL in 100 *μ*L of the suitable media were seeded into a 96-well microtiter plate and incubated for 24 h. The next day, 0.85 *μ*g/ml of AgNPs-PVP and AgNO_3_ and 500 *μ*g/ml of PVP were added to the cells and incubated overnight at 37°C with 5% CO_2_. After incubation, the cells were washed in PBS and lysed using the lysing buffer, and 100 *μ*l of cell lysate used for the ELISA test using human TNF-*α* and IL6 ELISA, as previously described [46, 47]. Briefly, the micro-ELISA plates were precoated with an antibody specific to human TNF-*α*/IL6 from kits obtained from Elabscience, USA, and incubated overnight. The next day, the ELISA plates were blocked with 4% FBS for 30 min, and 100 *μ*l samples/standards were added and incubated for 2 h. After washing, biotinylated detection antibodies specific for human TNF-*α*/IL6 were added and incubated for 1 h, followed by washing, adding an Avidin-Horseradish Peroxidase (HRP) conjugate to each well, and incubation for 30 min. Finally, the reaction was stopped by adding H_2_SO_4_, and the optical density of the developed colors was measured by an absorbance microplate reader (BioTek, Winooski, VT, USA). at 450 nm to determine the quantities of TNF-*α*/IL6 in the samples against a standard curve.

RETRACTED

### 2.8. Statistical Analysis

A statistical analysis was performed using a one-way analysis of variance (ANOVA). Minitab 16 Statistical Software with Tukey's multiple evaluations was used to compare the preparations. Statistically significant variances were approved when ^*∗*^*p* ≤ 0.05. ^*∗*^*p* < 0.05, ^*∗∗*^*p* < 0.01, or ^*∗∗∗*^*p* < 0.001 was considered statistically significant. All values are expressed as a mean ± standard deviation [10, 48].

## 3. Results

### 3.1. Silver Nanoparticles Preparation

AgNPs stabilized with PVP were efficiently prepared using the adopted procedures. After approximately 30 min of heating, the AgNO_3_ solution was completely reduced to silver nanoparticles, as indicated by the solution color change within 20 min. Hence, the influential role of PVP as a reducing polymer in silver nitrate solution. In addition, it was noticed that the prepared AgNPs-PVP did not show any precipitation or aggregation after their preparation, which also indicated the stabilizing action of PVP on the produced AgNPs.

### 3.2. Silver Nanoparticles Characterization

#### 3.2.1. Percentage Yield of AgNPs-PVP

ICP-OES results showed a high yield of the produced AgNPs-PVP of approximately 88.18 ± 15.8%. Silver cation concentrations in silver nitrate solution and in AgNPs-PVP were 550.8 ± 22.5 and 485.2 ± 30.5 *μ*M, respectively, which were considered the initial silver cations and silver cations in AgNPs concentrations.

RETRACTED

#### 3.2.2. UV-VIS Spectroscopy

Figure 1 shows the UV-VIS absorption spectra for AgNPs-PVP. Nanoparticles showed a strong absorption of electromagnetic waves in the visible region as a result of the surface plasmon resonance effect. The UV-VIS spectra showed a maximum wavelength at *λ*_max_ of 420 nm, which indicated the efficient nanoparticle preparation as well as spherical particle morphology [49, 50].

#### 3.2.3. FT-IR Spectroscopy

Figure 2 shows the FT-IR spectra for AgNO_3_, PVP, and AgNPs-PVP. The PVP trace (*A*) showed characteristic FT-IR bands of PVP presented in the carbonyl group of the pyrrolidone ring stretching vibration at 1634.52 cm^−1^, bending vibration at 1469.69, and 1384 cm^−1^ assigned to -CH deformation modes from -CH_2_. In addition, broadband located at 3449.90 cm^−1^ is related to the -OH stretching vibration [51]. AgNO_3_ spectra (trace B) showed several peaks around 3430.00, 2082.50, and 1633.52 cm^−1^. However, after the reduction of silver with the formation of AgNPs-PVP, it was also noted that the carbonyl peak of PVP was shifted from 1634.52 to 1636.30 (trace C). This shift was also reported by other investigators [51]. It could also be observed from the spectra of AgNPs-PVP (trace C) that the absence of the peaks of AgNO_3_ and the concomitant presence of the peaks of PVP confirmed the reduction and coating of silver with PVP and the formation of AgNPs-coated polymers. A similar result was also observed by other researchers, who concluded the absent peaks of AgNO_3_ in AgNPs confirmed the reduction of silver ions due to the reduction of capping material [52].

#### 3.2.4. Transmission Electron Microscope

AgNPs appeared as spherical nonaggregated particles with a mean size of 21.17 ± 0.8 nm as shown in Figure 3. The observed size was less than that calculated from DLS measurements, which was already recorded and demonstrated in similar studies [42, 53, 54]. Generally, DLS-based measurements depend on the hydrodynamic diameter; however, TEM-recorded size depends on the metal core of the nanoparticles [54].

#### 3.2.5. Size and Charge

DLS measurements showed that the prepared AgNPs-PVP had a size of 122.33 ± 17.61 nm with a polydispersity index of 0.49 ± 0.07. Furthermore, the nanoparticles produced had a negative charge of −19.23 ± 0.61 mV.

### 3.3. Physical Stability

A stability study against particle agglomerations and aggregations was performed at two different storage conditions. Generally, DLS measurements could be a useful technique to monitor the size and aggregate-related physical stability of nanoparticles [55]. Results revealed that particles remain intact in their size, charge, and shape when stored in the fridge at 4.0 ± 0.5°C. Size and charge were 123.35 ± 3.21 nm and −17.56 ± 3.8 mV, respectively, which showed a nonsignificant change (*p* ≥ 0.05; ANOVA/Tukey) compared with the freshly prepared particles. However, particles stored at room temperature showed a significant difference in size and charge (*p* < 0.05; ANOVA/Tukey).

RETRACTED

### 3.4. *In vitro* Anticancer Activity

The *in vitro* cytotoxicity of AgNO_3_, PVP, and AgNPs/PVP was investigated in PC3 using an MTT assay after 24 h of incubation. The cells were exposed to concentrations of 0.4–100 *μ*g/ml of AgNO_3_ & AgNPs/PVP and 0.5–5000 *μ*g/ml of PVP. Cells without sample administration were utilized as a control group for 100% cell viability. The anticancer activity increases as the concentration of the AgNPs-PVP increases compared to that of Ag ions (Figure 4). Meanwhile, the cytotoxicity of AgNO_3_ and AgNPs-PVP was evaluated against noncancerous cell lines, HSF, and cancerous cell lines, PC3. The cell monolayers were treated with concentrations of 0.4–100 *μ*g/ml of AgNO_3_ and AgNPs-PVP. As observed in Figure 4(a), the viability of HSF cells was affected upon treatment with higher concentrations of AgNO_3_ and AgNPs-PVP. The IC_50_ values were 62.61 ± 3.18 and 7.47 ± 0.38 for AgNO_3_ and AgNPs-PVP, respectively. Similar to PC3 cultures, AgNO_3_ and AgNPs-PVP decreased the cell viability of HSF, though in a way less than that observed in PC3 cells from these formulations. Interestingly, the inhibitory effect of AgNPs-PVP on PC3 was significantly more than what was observed on HSF. Moreover, the results showed also a significant reduction in the % viability (^*∗∗*^*p*  <  0.01) for AgNPs-PVP at concentrations of (0.4 and 1.6 *μ*g/ml), and ^*∗*^*p* < 0.05 at concentrations (6.3 and 25 *μ*g/ml) on PC3 cells compared with the same formula on the HSF cells noncancerous cells, indicating that the AgNPs-PVP have anticancerous effect (Figure 4(a)). The viability of HSF and PC3 cell lines was affected upon treatment with a higher concentration of PVP with an IC_50_ value of 1773 ± SD, which indicates the relative safety of PVP on noncancerous and cancerous cells (Figure 4(b)).

### 3.5. TNF-*α* Expression

In the next step, the effect of the AgNO_3_, PVP, and AgNPs-PVP on the expression of TNF-*α* in HSF and PC3 using ELISA assay was investigated. The results showed that the PC3 cells treated with AgNPs-PVP had a lower TNF-*α* with a significant value (^*∗*^*p* < 0.05) when compared with control cells, the value reached 16.84 ± 0.71 pg/ml versus 20.81 ± 0.44 pg/ml; respectively. Interestingly, the contrary was found in HSF cells, the TNF-*α* level showed nonsignificant data and increased to 21.42 ± 1.2 pg/ml in the cells treated with AgNPs-PVP compared to control cells, which was 18.83 ± 0.23 Pg/ml. These results confirmed that the AgNPs-PVP is more effective and has anti-TNF-*α* expression in cancerous cells than that obtained in noncancerous cells (Figure 5).

RETRACTED

### 3.6. IL-6 Expression

IL-6 as an inflammatory cytokine was measured as described in the material and methods section. It is clear from Figure 6 that HSF control cells showed production of 627.07 ± 9.22, 34.27 ± 1.2, 291.86 ± 3.22, and 4.93 ± 1.23 for control HSF cells and cells treated with PVP K25, AgNO_3_, and AgNPs-PVP, respectively. The HSF cells showed a highly significant level of reduction (^*∗∗∗*^*p* < 0.001) in IL-6 production. Moreover, the cancerous cells PC3 recorded a production of IL-6 of 73.48 ± 2.12, 82.78 ± 1.25, 60.32 ± 0.987, and 7.4 ± 0.99 for the control cells and cells treated with PVP K25, AgNO_3_, and AgNPs-PVP, respectively. Treatment of PC3 cells with AgNPs-PVP showed a higher level of reduction of IL-6 when compared with PC3 control cells. The IL-6 level showed a high reduction (^*∗∗*^*p* < 0.01) when treated with AgNPs-PVP. The value was reduced from 73.48 ± 2.1 pg/ml to 7.4 ± 0.99 pg/ml, respectively.

## 4. Discussion

The effect of different polymeric materials in producing stabilized AgNPs was studied, efficiently investigated, and discussed in our research group [28]. In this study, PVP with its negative charges could also interact with silver cations in silver nitrate solution, facilitating nanoparticle preparation and increasing the particle's stability in the aggregations [56, 57]. The coordination of silver ions with nitrogen and or oxygen atoms from PVP plays a fundamental role in nanoparticle formation [58]. It has been also discussed the protective role of PVP on AgNPs from growing and agglomeration [59]. Moreover, the successful preparation of AgNPs stabilized with PVP using the thermal method was also investigated [60]. The effective role of polymers as a potent reducing agent and stabilizing action on the produced nanoparticles was also studied by other researchers utilizing polymers like methylcellulose, ethyl cellulose, hydroxypropyl methylcellulose, and polyethylene glycol [28]. ICP efficiently recorded the amounts of silver cations in both silver nitrate solution and the prepared AgNPs-PVP. It was noticed that there is some loss in silver cations, which could be possibly related to the adsorption of Ag^+^ or AgNPs by the centrifuge tubes or pipettes, volume loss, or transportation during sample transfer for dilution and estimation [39]. The UV-VIS spectrum verified the successful preparation of AgNPs. The produced spectrum was also confirmed by other researchers [60]. In addition, asymmetrical particle size distribution could also be expected due to the presence of one absorption nanoparticle band, as noticed from the UV-VIS spectra in Figure 1 [61, 62]. Regarding the FT-IR analysis, the slight shift in wavenumbers for C=O absorption may result from bond weakening due to back bonding via partial donation of lone pair electrons from oxygen in PVP to the vacant orbital of silver. PVP has C-N and C=O bonds due to functional groups in its individual unit. It is reported that these groups have an affinity for silver ions and metallic silver coordination due to the N and O atoms in the polymer molecule [63]. Such coordination depends on the produced particle size; large particles are at the micron level, and the nitrogen group of heterocyclic rings of PVP is strongly bound to the carbonyl group [64, 65]. However, this observation is reversed in the nano-sized range, leaving the carbonyl and nitrogen free to coordinate with the silver metal [66]. The size and charge indicated the stability of the produced nanoparticles as well as a relatively narrow size distribution of particles as investigated by other researchers [67]. Similar results were also obtained from Ahlberg et al., who demonstrated the preparation of AgNPs capped with PVP with a hydrodynamic size of 120 nm and charge of −20 mV [67]. The produced negative charge also delineates the formation of the coating layer of PVP around the formed nanoparticles. Negatively charged particles are useful particles in terms of interaction with positively charged bacteria as well as could interact with some targeting moieties like somatostatin, which have a positive charge for active targeting in different types of cancer [68]. AgNPs showed maximum physical stability at low temperatures, compared with high storage temperature conditions. Particles showed aggregation, and about 3-4 particles were attracted together to get a final size of 415.66 ± 34.03 nm and a charge of −11.03 ± 2.5 mV. Such an observation was also recorded in our previous study [28]. In addition, lowering the value of the zeta potential demonstrated the formation of particle aggregates. Similarly, Cheng et al. [69] demonstrated the formation of particle aggregates of AgNPs stabilized with chondroitin sulfate when stored at room temperature after 21 days.

RETRACTED

The inhibitory effect of AgNPs-PVP on PC3 cell lines was significantly more than what was observed on HSF. Moreover, the results also showed a significant reduction in the % viability (^*∗∗*^*p* < 0.01) for AgNPs-PVP at the used concentrations of (0.4 and 1.6 *μ*g/ml), and ^*∗*^*p* < 0.05 at concentrations (6.3 and 25 *μ*g/ml) on PC3 cells compared with the same formula on the HSF noncancerous cells, indicating that the AgNPs-PVP have an anticancerous effect. This can be explained, as the cancer cell being more sensitive to the concentration of Ag^0^ than the noncancerous cell [18]. Moreover, this superior inhibition might be associated with the presence of AgNPs in a polymeric film. The cell proliferation was stopped due to Ag^0^ in AgNPs-PVP. AgNPs-PVP showed significant reductions (^*∗*^*p* ≤ 0.05) in cell proliferation when treated with AgNPs-PVP treatment. The cells showed a decrease in % viability, meaning that the higher concentrations of AgNPs-PVP and Ag ions have more proliferation on PC3 cells. Furthermore, a higher reduction in the cell viability indicated that the AgNPs-PVP have a selective action on the cancer cells PC3 compared with normal HSF cells. It was reported that AgNO_3_ also has a degree of proliferation significantly due to the increased concentration of Ag^0^. These findings prove that AgNPs-PVP cause cytotoxicity inside the cells by releasing the Ag ions [70]. These conclusions agreed with those reported by Krishnaraj et al. [71], who proved that AgNO_3_ and HAuCl_4_ both have cytotoxic activity against human breast cancer cells (MDA-MB-231). Our findings also delineate the significance of the prepared formulation towards prostate cancer cells, presented with a lower IC_50%_ compared with the previously published work. Prasannaraj et al. showed a higher IC_50%value_ forPC-3 cell lines using AgNPs produced with different plant extracts acting as a reducing and capping agent [72]. Another study showed a higher IC_50%_ of AgNPs of around173.21 *μ*g/ml using PC-3 cell lines, compared with our obtained data [73]. Chitosan/poly (vinyl alcohol) blend doped with AgNPs showed an IC_50%_ of 23.1 *μ*g/ml against PC-3 cell lines, which is also higher than that obtained from the prepared AgNPs-PVP [16]. A recent study performed by Anwar et al. demonstrated IC_50%_ values of 38 and 34 *μ*g/ml for *Caralluma tuberculata* capped AgNPs and *Caralluma tuberculata* capped AgNPs hybridized with poly(ethylene glycol) methacrylate, respectively using PC-3 cell lines [74].

The synthesized AgNPs-PVP can affect cells and cause a significant decrease in (TNF-*α*, and mRNA) levels. AgNPs-PVP significantly (^*∗*^*p* < 0.05) reduced TNF-*α* production in the cultured PC3 compared with the noncancerous HSF cells. This result showed a significant decrease in TNF production, which was not the case in noncancerous cells and untreated PC3 cells. These findings suggested that AgNPs-PVP may be a possible therapeutic target for PC3 cells (prostate cancer). The Ag ions in AgNPs-PVP were proved to have a higher cell internalization, which accounts for the observed inhibitory effects on PC3 cell line differentiation at higher NPs concentrations [70]. TNF-*α* is a strong inflammatory cytokine that has been shown to influence immunological homeostasis, inflammation, apoptosis, proliferation, and tumor invasion, all of which could be considerably reduced by the AgNPs-PVP [75, 76].

RETRACTED

In this study, it was proved that AgNPs-PVP has a powerful reduction of IL-6. The results showed a significant decrease of IL-6 (^*∗∗*^*p* < 0.01) in the case of cancerous cells PC3, confirming that the AgNPs-PVP could reduce the inflammatory mediator in the case of cancer. This finding could be a promising result as a synergistic effect of AgNPs-PVP against TNF-*α* and IL-6. Furthermore, our findings showed the powerful effect of AgNPs-PVP in noncancerous cells, which showed highly significant results (^*∗∗∗*^*p* < 0.001). Since HSF cells showed a reduction in the production of IL-6 from 627.07 ± 9.22 to 4.93 ± 1.23 when the HSF cells were treated with AgNPs-PVP, respectively. The HSF cells showed a high level of reduction (^*∗∗∗*^*p* < 0.001) in IL-6 production. The obtained results agreed with those reported by Parnsamut and Brimson [77], who stated that each leukemic cell line treated with nanoparticles demonstrated a different signaling pathway response, which either inhibited or stimulated cytokine production, resulting in an anticell proliferation in the laboratory. A considerable impact on leukemia treatment may be expected in the future due to the effects of AgNPs and AuNPs on leukemic cell lines.

Based on the current findings, AgNPs-PVP exhibit anticancer activity against PC3 compared to HSF. Similar results were obtained from previous work [17, 18, 67]. (Firdhouse and Lalitha). PVP as a stabilizer for AgNPs allows the nanosilver to interact more closely with cancer cells and liberate efficiently into the cytoplasm to enhance Ag ions pharmacological effects. In addition, AgNPs-PVP exhibited higher anticancer activity against prostate cancer cells compared to AgNO_3_. This indicates the recruitment of AgNPs-PVP may decrease the concentrations required to produce an antitumor effect. In addition, PVP might play a part in the toxicity of AgNPs. The current study confirmed that AgNPs-PVP inhibits PC3 viability at concentrations of 0.4 *μ*g/ml and more. The cellular internalization of the AgNPs is mainly caused by endocytosis. The acidity of the endolysosome increases the release of Ag ions from AgNPs. These reactive ions decrease protease activity, leading to blocking the autophagic response. This action results in disturbances in cellular homeostasis, leading to programmed cell death [17, 18]. The inhibitory action of AgNPs is referred to as the “Trojan-horse”-type mechanism in which the cytotoxic activity emerges only after the cellular uptake. In addition, the decrease in proliferation is due to a reduction in energy and hypoxia, resulting from stimulation of AMPK/mTOR signaling [18]. Previous work reported that exposure to AgNPs even at low concentrations could reduce ATP generation in many cancer cells and cause cell death. Another study revealed that hypoxia contributes to autophagy activation in lung cancer cells when treated with AgNPs [67]. Further studies are needed to assess the role of the PVP polymeric coat of AgNPs/PVP in the inhibition of other cancer cell proliferation.

RETRACTED

## 5. Conclusions

AgNPs-PVP was efficiently prepared and showed higher physical stability upon reducing a silver nitrate solution with PVP. In addition, PVP formed an efficient coat around the formed NPs, as demonstrated by the FT-IR study and zeta potential value. AgNPs-PVP retains its physical stability at a lower temperature compared with storage at high-temperature conditions. The produced AgNPs-PVP showed significant anticancer activity against PC3 cell lines, which was confirmed in secondary tests based on the IL-6 and TNF-alpha levels in HSF, and PC3 cells. AgNPs-PVP showed a promising nanoformulation for efficient targeting of prostate cancer.

## Figures and Tables

**Figure 1:** The UV absorption spectrum of AgNPs-PVP. The spectrum showed a maximum wavelength at *λ*_max_ of 420 nm.

**Figure 2:** FT-IR spectra of PVP K-25 (a); silver nitrate (b); and AgNPs-PVP (c).

**Figure 3:** Transmission electron microscope images of AgNPs-PVP. Scale bar represents 100 nm and magnification 50000×. Image B shows the size of the produced AgNPs-PVP, with a mean diameter of 21.17 ± 0.8 nm.

**Figure 4:** Cell viability of PC3 and HSF cells after incubation for 24 h at 37°C with different concentrations of AgNO_3_, AgNPs-PVP (a), and PVP K25 (b). As controls, the medium was used, all tests were conducted in triplicate, the data are shown as the mean ± standard deviation, and they are presented in (%) of the control. ^*∗*^*p* < 0.05, and ^*∗∗*^*p* < 0.01 were considered statistically significant.

**Figure 5:** Determination of TNF-*α* in PC3 (prostate cancer), HSF (normal cells), for AgNPs-PVP, PVP K25, and AgNO_3_.

**Figure 6:** Determination of IL-6 production for AgNPs-PVP, PVP, and AgNO_3_ performed on normal cell (HSF) and cancer cell lines (PC3), concentrations (pg/ml).

## Data Availability

The data used to support the findings of this study are included within the article.
